The article "Comparison of the Effects of Hysteroscopic Cold Broad Sword Play Combined with Estrogen and Progestin Sequential Therapy and Drospirenone and Ethinylestradiol Tablets in Patients with Severe Intrauterine Adhesion" was retracted in 2023. Reasons: signs of a paper mill; suspected computer-generated content; unreliable results or conclusions; lack of ethics approval or compliance.

# Comparison of the Effects of Hysteroscopic Cold Broad Sword Play Combined with Estrogen and Progestin Sequential Therapy and Drospirenone and Ethinylestradiol Tablets in Patients with Severe Intrauterine Adhesion

**DOI:** 10.1155/2022/9898228

**Published:** 2022-07-31

**Authors:** Liping Zhou, Liqin Zhou, Tingting Wang

**Affiliations:** ^1^Department of Gynecology, Zhuji People's Hospital of Zhejiang Province, Zhuji, Zhejiang 311800, China; ^2^Department of Pharmacy, Zhuji People's Hospital of Zhejiang Province, Zhuji, Zhejiang 311800, China; ^3^Department Obsterics and Gynecology, Zhuji Maternal and Child Health Hospital, Zhuji, Zhejiang 311800, China

## Abstract

**Objective:**

To compare the effects of hysteroscopic cold broad sword play combined with estrogen and progestin sequential therapy and drospirenone and ethinylestradiol tablets in patients with severe intrauterine adhesion.

**Methods:**

One hundred and eight patients with severe IUA admitted to our hospital from May 2019 to October 2021 were selected for the study. Patients were divided according to their treatment regimen into group A (*n* = 54) treated with hysteroscopic cold broad sword play + drospirenone and ethinylestradiol tablets and group B (*n* = 54) treated with hysteroscopic cold broad sword play + estrogen and progestin sequential therapy. The two groups were compared in terms of perioperative indicators, recovery of uterine cavity status, inflammatory factor (C-reactive protein (CRP), interleukin 6 (IL-6), and interleukin 8 (IL-8)] levels), World Health Organization Quality of Life Brief Scale (WHOQOL-BREF) score, and clinical outcome at 3 months postoperatively.

**Result:**

After surgery, the duration of abdominal pain and vaginal bleeding was shorter in group A than in group B (*P* < 0.05). After surgery, the time of menstruation return was shorter in group A than in group B, and the menstrual flow score was higher than in group B (*P* < 0.05). At 3 months after the surgery, the uterine blood flow index, endometrial thickness, and uterine cavity volume were higher in group A than in group B, and the number of uterine readhesion was lower than in group B (*P* < 0.05). 3 months after the surgery, the CRP, IL-6, and IL-8 levels decreased in both groups and were lower in group A than in group B (*P* < 0.05). At 3 months after the surgery, the WHOQOL-BREF scores for each indicator were higher in both groups than before surgery and were higher in group A than in group B (*P* < 0.05). At 3 months after the surgery, the overall valid rate of group A was 94.44% better than that of group B at 79.63% (*P* < 0.05).

**Conclusion:**

The combination of hysteroscopic cold broad sword play with drospirenone and ethinylestradiol tablets has been shown to be more effective than combined estrogen and progestin sequential therapy in the treatment of patients with severe IUA, which significantly improves the post-operative menstrual status and uterine cavity morphology, significantly reduces the level of inflammatory factors in the patient's body, and significantly improves the quality of life, which is of value.

The article "Comparison of the Effects of Hysteroscopic Cold Broad Sword Play Combined with Estrogen and Progestin Sequential Therapy and Drospirenone and Ethinylestradiol Tablets in Patients with Severe Intrauterine Adhesion" was retracted in 2023. Reasons: signs of a paper mill; suspected computer-generated content; unreliable results or conclusions; lack of ethics approval or compliance.

## 1. Introduction

Intrauterine adhesion (IUA), also known as Asherman's syndrome, can be triggered by any intrauterine operation that may cause damage to the endometrium, with painless abortion being the main cause, and its incidence has increased in recent years. The disease refers to the damage of the basal layer of the human endometrium, the destruction of the proliferation and secretion functions of the endometrium, and the partial or complete closure of the uterine cavity [1, 2]. Patients may suffer from abnormal menstruation, placenta praevia, miscarriage, and infertility, which seriously affect their physical and mental health and quality of life [3–5]. To restore the uterine lining to normal, hysteroscopic surgery is clinically indicated. The two main surgical procedures are hysteroscopic electrosurgery and hysteroscopic cold broad sword play, which have different results. Of these, the former can effectively separate, excise, and stop bleeding at the site of uterine adhesions and is the preferred option for the treatment of uterine adhesions, but the electrothermal effect produced during electrodes separation of adhesions tends to reinjure the human endometrium, causing postoperative uterine readhesions to occur with a recurrence rate of up to 15% or more [6]. Hysteroscopic cold broad sword play is a new separation technique that has been used in recent years to treat IUAs. It belongs to the category of nonenergy instruments. Different microscissors can be selected according to the adhesion status of different parts, such as the uterine floor, uterine body, and uterine angle, to give full play to the best separation effect, which provides the possibility for the effective separation of adhesion in patients with moderate and severe IUA. It also has the characteristics of a high one-time success rate, rapid postoperative menstrual recovery, and a high pregnancy rate [7]. In addition to this, it is essential to provide complementary treatment after the operation for uterine adhesions. The intrauterine device (IUD) is a contraceptive device placed in the uterine cavity. In recent years, our hospital has mostly adopted the method of placing birth control rings during the operation to achieve the role of physical isolation and prevent readhesion, which can be effective. However, the study [8] showed that patients with severe uterine adhesions have a slow postoperative recovery due to the extensive and invasive nature of the procedure. Although an intraoperative birth control ring can be placed, its isolation area is limited and does not completely separate the anterior and posterior walls of the uterus, and patients remain at a greater risk of postoperative readhesions. Since then, it has been suggested that the combination of postoperative manual cycle therapy may reduce the risk of readhesion in patients, but the stability of its effect and the safety of long-term application of these preventive methods are controversial. Drospirenone and ethinylestradiol tablets are a fourth-generation combination oral contraceptive, the main ingredients of which are drospirenone and ethinylestradiol. In recent years, studies have shown that oral drospirenone and ethinylestradiol tablets have a good preventive effect on IUA after cervical cleansing. Based on the above, this study intends to compare the efficacy of estrogen and progestin sequential therapy and drospirenone and ethinylestradiol tablet therapy after intrauterine adhesions decomposition in order to obtain the best medication scheme to prevent readhesions after intrauterine adhesions decomposition.

The article "Comparison of the Effects of Hysteroscopic Cold Broad Sword Play Combined with Estrogen and Progestin Sequential Therapy and Drospirenone and Ethinylestradiol Tablets in Patients with Severe Intrauterine Adhesion" was retracted in 2023. Reasons: signs of a paper mill; suspected computer-generated content; unreliable results or conclusions; lack of ethics approval or compliance.

## 2. Materials and Methods

### 2.1. General Data

One hundred and eight patients with severe IUA admitted to our hospital from May 2019 to October 2021 were selected for the study. Patients were divided according to their treatment regimen into group A (*n* = 54) treated with hysteroscopic cold broad sword play + drospirenone and ethinylestradiol tablets and group B (*n* = 54) treated with hysteroscopic cold broad sword play + estrogen and progestin sequential therapy. The baseline data of the two groups are shown in Table 1; all differences were not statistically significant (*P* > 0.05) and were comparable.

### 2.2. Inclusion and Exclusion Criteria

Inclusion criteria were defined as follows: ① IUA diagnosis referred to the Chinese Expert Consensus on Clinical Management of Uterine Adhesions [9]; ②diagnosis of IUA confirmed by 3D ultrasound and hysteroscopy; ③those with complete clinical information; ④diagnosis of severe IUA according to March's classification; ⑤those who met the indications for hysteroscopic cold broad sword play treatment and underwent the procedure in our hospital; and ⑥combined with psychiatric illness and unable to cooperate with the researcher.

Exclusion criteria were defined as follows: ①Coagulation disorders; ②contraindicated for hysteroscopic surgery; ③combination of serious infectious diseases; ④malformations of the reproductive system; ⑤combined with other reproductive disorders; and ⑥combined with other reproductive disorders.

The article "Comparison of the Effects of Hysteroscopic Cold Broad Sword Play Combined with Estrogen and Progestin Sequential Therapy and Drospirenone and Ethinylestradiol Tablets in Patients with Severe Intrauterine Adhesion" was retracted in 2023. Reasons: signs of a paper mill; suspected computer-generated content; unreliable results or conclusions; lack of ethics approval or compliance.

### 2.3. Methods

Patients in both groups were treated with hysteroscopic cold broad sword play.

Preoperative preparation: on admission, a detailed history of the uterine cavity disease and surgery was obtained and all gynaecological, internal, and preoperative ancillary investigations were completed. The surgery was performed 3 to 7 days after menstruation. All patients were given misoprostol (China Resources Zizhu Pharmaceutical Co., Ltd., approval No.: H20000668, specification: 0.2 mg) 0.2 mg orally at bedtime 1 night before the surgery and abstained from drinking and eating for 6 hours before the surgery. 25 *μ*g of misoprostol vaginal tablets (Guangzhou Langsheng Pharmaceutical Co., Ltd., approval No.: H20203249, specification: 25 *μ*g)were placed vaginally 3 hours before the surgery to soften and dilate the cervix. All patients were placed in a bladder lithotomy position, intravenous total inebriation was performed, and the vagina was routinely disinfected. The cervix was exposed with a speculum, and a hysteroscope was placed under ultrasound guidance. Surgical treatment was carried out after identifying the intrauterine adhesions.

Intraoperative operations: microscissors were inserted through the instrument hole and the type of scissors was selected according to the site of adhesions. The adhesive band was cut and the scar tissue was removed and an IUD (T-ring) was placed at the same time and postoperative balloon compression was applied to stop bleeding.

Postoperative treatment: both groups were routinely treated with antibiotics for 3 days after the operation. On top of this, group A was treated with drospirenone and ethinylestradiol tablets (Bayer Weimar GmbH and Co. KG, approval No.: J20171071, specification: drospirenone 3 mg + ethinylestradiol 0.03 mg) orally on the day of surgery, 1 tablet/day for 21 days, stopping for 7 days before starting the second cycle of treatment for 3 cycles; group B was treated with estrogen and progestin sequential therapy on the day of surgery, i.e. estradiol valerate (Peking Union Pharmaceuticals, approval No.: H20000031, specification: 0.5 mg) orally, 2 mg/dose, 2 times/day for 21 days, on the 11th day with the addition of dydrogesterone tablets (Abbott Biologicals B. V., approval No.: H20170221, specification: 10 mg), orally, 10 mg/dose, 2 times/day, stopping after day 21 for 7 days before starting the next cycle of treatment, 3 cycles of treatment. All patients finished treatment in the 3rd month after the procedure and returned to the hospital 3–7 days after menstruation for a follow-up hysteroscopy and removal of the IUD.

The article "Comparison of the Effects of Hysteroscopic Cold Broad Sword Play Combined with Estrogen and Progestin Sequential Therapy and Drospirenone and Ethinylestradiol Tablets in Patients with Severe Intrauterine Adhesion" was retracted in 2023. Reasons: signs of a paper mill; suspected computer-generated content; unreliable results or conclusions; lack of ethics approval or compliance.

### 2.4. Observed Indicators

1. Record the duration of abdominal pain and vaginal bleeding after surgery for patients in groups A and B.
2. Record the time of menstruation return and menstrual flow score after surgery in groups A and B. The latter was assessed on the basis of a score based on the product of the area of menstrual blood stained and the size of the clot. Bloodstained area <1/3 of sanitary napkin, 1/3 to 3/5 of sanitary napkin, and >3/5 of sanitary napkin were counted as 1, 5, and 20 points, respectively, 1, 3, and 5 marks for blood clot size <1 yuan coin, = 1 yuan coin, > 1 yuan coin, respectively. The total score was 1 ∼ 100. The higher the score, the greater the amount of menstruation [10].
3. Record the status of the uterine cavity at the 3-month postoperative follow-up of patients in groups A and B. Vaginal 3D ultrasound was used to detect uterine blood flow index, endometrial thickness, and uterine cavity volume. The criteria for determining uterine readhesion were based on the March classification: absence of adhesions: no adherent tissue was seen at hysteroscopy; mild adhesions: adhesions covering ≤1/4 of the uterine cavity, or only membranous adhesions, with no or only minor adhesions at the tubal orifice and fundus seen microscopically; moderate adhesions: adhesions ranging from 1/4 to 3/4 of the uterine cavity, no adhesions between the uterine walls, hysteroscopic view of the opening of the fallopian tube and partial atresia of the upper uterine cavity; severe adhesions: adhesions >3/4 of the uterine cavity, atresia at the opening of the fallopian tube, and the upper part of the fundus [11].
4. Measure inflammatory factor levels of patients in groups A and B before and 3 months after the surgery. The main tests were for C-reactive protein (CRP), interleukin 6 (IL-6), and interleukin 8 (IL-8). The assays were all enzyme-linked immunosorbent assays and the kits were purchased from Shanghai Sango Biotechnology Co.
5. Record the WHOQOL-BREF scores of patients in groups A and B before and 3 months after the surgery. The WHO Quality of Life Brief Scale (WHOQOL-BREF) was used to assess the quality of life, which consists of four items: physical, psychological, environmental, and social relationships, with individual scores ranging from 0 to 100, and the scores are directly proportional to the quality of life [12].
6. Assess the clinical outcome of patients in groups A and B at 3 months after the surgery. Assessment criteria: the patients were healed when the morphology and size of the uterine cavity returned to normal; the opening of the fallopian tubes was seen bilaterally and the menstrual cycle and menstrual flow returned to normal; the patients were valid if the morphology and size of the uterine cavity were basically normal; the opening of the fallopian tubes could not be expressed bilaterally and the menstrual cycle was restored but the menstrual flow was low; failure to meet the criteria for effectiveness was considered ineffective. Total effective rate = the sum of the ratio of healed to valid.

The article "Comparison of the Effects of Hysteroscopic Cold Broad Sword Play Combined with Estrogen and Progestin Sequential Therapy and Drospirenone and Ethinylestradiol Tablets in Patients with Severe Intrauterine Adhesion" was retracted in 2023. Reasons: signs of a paper mill; suspected computer-generated content; unreliable results or conclusions; lack of ethics approval or compliance.

### 2.5. Statistical Methods

SPSS 22.0 software was applied, and the measurement data were expressed as mean ± standard deviation and compared by *t*-test. Count data were expressed as ratios, and the *χ*^2^ test was used for comparison. *P* < 0.05 was considered statistically significant.

## 3. Results

### 3.1. Comparison of the Duration of Abdominal Pain and Vaginal Bleeding after Surgery in Groups A and B

After the surgery, the duration of abdominal pain and vaginal bleeding were shorter in group A than in group B. The difference was statistically significant (*P* < 0.05) (Figures 1 and 2).

### 3.2. Comparison of Time of Menstruation Return and Menstrual Flow Score after Surgery in Groups A and B

After the surgery, the time of menstruation return was shorter in group A than in group B, and the menstrual flow score was higher than in group B. The differences were all statistically significant (*P* < 0.05) (Figures 3 and 4).

### 3.3. Comparison of the Uterine Cavity Status at 3 Months after Surgery in Groups A and B

3 months after the surgery, the uterine blood flow index, endometrial thickness, and uterine cavity volume were higher in group A than in group B, and the number of uterine readhesions was lower than in group B. The difference was statistically significant (*P* < 0.05) (Figures 5–8).

### 3.4. Comparison of Inflammatory Factors Levels before and after Surgery in Groups A and B

3 months after the surgery, the CRP, IL-6, and IL-8 levels decreased in both the groups and were lower in group A than in group B, and the difference was statistically significant (*P* < 0.05) (Figures 9 and 10).

### 3.5. Comparison of WHOQOL-BREF Scores before and after Surgery in Groups A and B

At 3 months after the surgery, the WHOQOL-BREF scores for each indicator were higher in both groups than before surgery and were higher in group A than in group B, and the difference was statistically significant (*P* < 0.05) (Figures 11 and 12).

### 3.6. Comparison of Clinical Efficacy in Groups A and B

At 3 months after the surgery, the overall validity rate of group A was 94.44% better than that of group B at 79.63%, and the difference was statistically significant (*P* < 0.05) (Table 2).

## 4. Discussion

Although with the development of medical imaging, the use of ultrasonography and hysteroscopy provides a visual and complete picture of the uterine cavity, and the IUA separation can be safely performed under hysteroscopy to separate the adherent tissue. However, some patients (especially those with severe IUA) still undergo a second operation at the time of postoperative review due to readhesions, which aggravates the physical and psychological damage and financial burden on the patient, while also reducing the patient's satisfaction with the treatment.

The article "Comparison of the Effects of Hysteroscopic Cold Broad Sword Play Combined with Estrogen and Progestin Sequential Therapy and Drospirenone and Ethinylestradiol Tablets in Patients with Severe Intrauterine Adhesion" was retracted in 2023. Reasons: signs of a paper mill; suspected computer-generated content; unreliable results or conclusions; lack of ethics approval or compliance.

The cold knife used in hysteroscopic cold broad sword play is free of electrothermal radiation, which can avoid endometrial damage, destruction, and scar formation caused by thermal radiation and can facilitate the recovery of the uterine cavity morphology [13, 14]. The intraoperative placement of the IUD can isolate the adhesive surface and open up the uterine cavity for the purpose of preventing a recurrence. The addition of postoperative estrogen and progestin sequential therapy promotes the growth of the patient's endometrium and interstitial cells, promotes the growth of blood vessels, mesenchyme, and glands in the basal layer of the endometrium, accelerates the thickening of the endometrial layer, and promotes rapid reepithelialisation of the wounds produced by surgical separation [15, 16]. One study [17] pointed out that in patients with severe IUA, given the severe damage to the basal endometrium, high doses of estrogen are required to stimulate endometrial proliferation after surgery, but the local hyperestrogenic environment may promote IUA and endometrial fibrosis by increasing serum levels of proadhesive and profibrotic cytokines such as transforming growth factor beta 1 (TGF-*β*1) and basic fibroblast growth factor (bFGF). As a result, the ability of the endometrium to regenerate is significantly reduced after severe damage to the basal layer of the endometrium, and the emphasis on high estrogen levels may be counterproductive. The present results show that patients in group B who were treated with postoperative estrogen and progestin sequential therapy had less favourable postoperative menstrual conditions and less rapid recovery of uterine morphology than patients in group A who were treated with drospirenone and ethinylestradiol tablets, and their postoperative IUA recurrence rate was higher than that of patients in group A. The reason for this may be due to the fact that surgery creates favourable conditions for the recovery of the patient's uterine cavity morphology. In addition to postoperative treatment with drospirenone and ethinylestradiol tablets, although the drug is short-lived, it is well absorbed and can reach blood concentration within a short period of time, inhibit ovulation and, at the same time, can play a powerful role in repairing the endometrium after separation of the uterine cavity adhesions, thus effectively shortening the duration of vaginal bleeding. The patient can resume menstruation as soon as possible after stopping the drug and form a new menstrual cycle. It can also effectively improve the cervical mucus viscosity and prevent the development of IUA as well as internal uterine infections. Compared to the estrogen and progestin sequential therapy, drospirenone and ethinylestradiol tablets are lower in ethinylestradiol and have fewer side effects, which ensures patient safety. A recent study [18] in patients with dysmenorrhoea found a significant reduction in the number and intensity of days of menstrual pain in patients treated with the ethinylestradiol (EE)/drospirenone (DRSP) regimen compared to sequential therapy. In this result, the duration of abdominal pain was shorter in group A patients than in group B after treatment. This suggests that the addition of drospirenone and ethinylestradiol tablet treatment after hysteroscopic cold broad sword play also had a significant effect on improving abdominal pain in patients with IUA.

The article "Comparison of the Effects of Hysteroscopic Cold Broad Sword Play Combined with Estrogen and Progestin Sequential Therapy and Drospirenone and Ethinylestradiol Tablets in Patients with Severe Intrauterine Adhesion" was retracted in 2023. Reasons: signs of a paper mill; suspected computer-generated content; unreliable results or conclusions; lack of ethics approval or compliance.

At 3 months after surgery, CRP, IL-6, and IL-8 levels decreased in both groups and were lower in group A than in group B. This suggests that postoperative treatment with drospirenone and ethinylestradiol tablets is better at repairing endometrial damage and reducing the level of inflammatory factors in the body than the addition of estrogen and progestin sequential therapy. Analysis of the reasons for the above results, drospirenone and ethinylestradiol tablets is composed of drospirenone and ethinylestradiol. Drospirenone is a 17*ɑ*-spirolactone derivative, similar to natural progesterone, with progestogenic activity, antiandrogenic activity, and antisalt corticosteroid activity. It antagonizes estrogen receptors, has a strong affinity for progesterone, induces atrophy of meconium tissue, helps to expel postoperative uterine residues, and also inhibits bacterial entry, reducing the incidence of genital infectious diseases such as pelvic inflammatory disease [19, 20]. At 3 months after surgery, the WHOQOL-BREF scores for each index were higher in both groups than before surgery, and the WHOQOL-BREF scores for each index and overall clinical validity rate were higher in Group A than in Group B. It is suggested that the addition of drospirenone and ethinylestradiol tablets after hysteroscopic cold broad sword play for patients with severe IUA may indirectly improve their quality of life by controlling their condition and accelerating their recovery.

The article "Comparison of the Effects of Hysteroscopic Cold Broad Sword Play Combined with Estrogen and Progestin Sequential Therapy and Drospirenone and Ethinylestradiol Tablets in Patients with Severe Intrauterine Adhesion" was retracted in 2023. Reasons: signs of a paper mill; suspected computer-generated content; unreliable results or conclusions; lack of ethics approval or compliance.

In short, the combination of hysteroscopic cold broad sword play with drospirenone and ethinylestradiol tablets has been shown to be more effective than combined estrogen and progestin sequential therapy in the treatment of patients with severe IUA, which significantly improves the postoperative menstrual status and uterine cavity morphology, significantly reduces the level of inflammatory factors in the patient's body, and significantly improves the quality of life, which is of value and has an application value. The treatment protocols used in this study have some drawbacks, as they do not completely prevent the occurrence of postoperative readhesions, and the development and application of relevant aspects still need further exploration.

## Figures and Tables

**Figure 1:** Duration of abdominal pain. *Note*. Δ indicates *P* < 0.005 for the difference between groups A and B.

**Figure 2:** Duration of vaginal bleeding. *Note*. Δ indicates *P* < 0.05 for the difference between groups A and B.

**Figure 3:** Time of menstruation return. *Note*. Δ indicates *P* < 0.005 for the difference between groups A and B.

**Figure 4:** Menstrual flow score. *Note*. Δ indicates *P* < 0.05 for the difference between groups A and B.

**Figure 5:** Uterine blood flow index.

**Figure 6:** Endometrial thickness.

**Figure 7:** Uterine cavity volume. *Note*. Δ indicates *P* < 0.05 for the difference between groups A and B.

**Figure 8:** Number of uterine readhesion. *Note*. Δ indicates *P* < 0.05 for the difference between groups A and B.

**Figure 9:** Inflammatory factors levels before surgery. *Note*. Δ indicates *P* < 0.005 for the difference between groups A and B.

**Figure 10:** Inflammatory factors levels 3 months after surgery. *Note*. Δ indicates *P* < 0.05 for the difference between groups A and B.

**Figure 11:** WHOQOL-BREF score before surgery.

**Figure 12:** WHOQOL-BREF score at 3 months after surgery. *Note*. Δ indicates *P* < 0.05 for the difference between groups A and B.

**Table 1:** Baseline information for groups A and B.

Items	Group A	Group B	*t*	*P*
Age (years)	31.41 ± 2.76	31.85 ± 2.56	0.859	0.392
BMI (kg/m^2^)	25.67 ± 1.70	25.69 ± 2.08	0.055	0.957
Disease duration (months)	5.11 ± 0.90	5.17 ± 0.84	0.358	0.721
Pregnancy (times)	2.57 ± 1.14	2.61 ± 0.76	0.215	0.831
Delivery (times)	1.46 ± 0.69	1.54 ± 0.61	0.638	0.525

**Table 2:** Clinical efficacy in groups A and B (*n*,%).

Groups	Healed	Valid	Invalid	Overall valid
Group A	33 (61.11)	18 (33.33)	3 (5.56)	51 (94.44)
Group B	30 (55.56)	13 (24.07)	11 (20.37)	43 (79.63)
*χ * ^2^	0.343	1.131	5.252	5.252
*P*	0.558	0.288	0.022	0.022

## Data Availability

The primary data to support the results of this study are available at reasonable request to the corresponding author.
